# Peritumor Edema Serves as an Independent Predictive Factor of Recurrence Patterns and Recurrence-Free Survival for High-Grade Glioma

This article has been retracted.

**DOI:** 10.1155/2022/9547166

**Published:** 2022-07-27

**Authors:** Jie Chen, Hui Qiu, Rui Chen, Jiani Huang, Liang Chen, Juncheng Wan, Qi Chen, Longzhen Zhang

**Affiliations:** ^1^School of Medical Imaging, Xuzhou Medical University, Xuzhou 221000, China; ^2^Department of Radiation Oncology, Affiliated Hospital of Xuzhou Medical University, Xuzhou 221000, China

## Abstract

**Objective:**

This study is aimed at analyzing the factors affecting the recurrence patterns and recurrence-free survival (RFS) of high-grade gliomas (HGG).

**Methods:**

Eligible patients admitted to the Affiliated Hospital of Xuzhou Medical University were selected. Subsequently, the effects of some clinical data including age, gender, WHO pathological grades, tumor site, tumor size, clinical treatments, and peritumoral edema (PTE) area and molecular markers (Ki-67, MGMT, IDH-1, and p53) on HGG patients' recurrence patterns and RFS were analyzed.

**Results:**

A total number of 77 patients were enrolled into this study. After analyzing all the cases, it was determined that tumor size and tumor site had a significant influence on the recurrent patterns of HGG, and PTE was an independent predict factor of recurrence patterns. Specifically, when the PTE was mild (<1 cm), the recurrence pattern tended to be local; in contrast, HGG was more likely to progress to marginal recurrence and distant recurrence. Furthermore, age and PTE were significantly associated with RFS; the median RFS of the population with PTE < 1 cm (23.60 months) was obviously longer than the population with PTE ≥ 1 cm (5.00 months).

**Conclusions:**

PTE is an independent predictor of recurrence patterns and RFS for HGG. Therefore, preoperative identification of PTE in HGG patients is crucially important, which is helpful to accurately estimate the recurrence pattern and RFS.

## 1. Introduction

Heterogeneous central nervous system (CNS) tumors account for about 80% of the primary malignancy in CNS [1]. Among them, high-grade gliomas (HGG), which are comprised primarily of World Health Organization (WHO) grade III anaplastic astrocytoma and WHO grade IV glioblastoma multiforme (GBM), possess strong invasive capability without obvious boundaries. Such characteristics make HGG difficult to be completely healed by operation, chemotherapy, radiotherapy, target therapy, and other treatments [2–4]. GBM as a kind of HGG accounts for about 25% of gliomas [5]. Generally, patients with HGG have poor prognosis owing to the high rate of recurrence in the short term [6]; the median overall survival (OS) of anaplastic astrocytoma patients is about 3 years [7], while that of GBM patients is less than 14 months [8]. The Chinese guidelines for the diagnosis and treatment of GBM in the CNS (2015) recommend the Stupp regimen proposed by the European Organization for Research and Treatment of Cancer as the first-line treatment option for Chinese patients with GBM [9]. However, after first-line treatment including surgery, radiotherapy, and temozolomide chemotherapy, the prognosis of GBM patients remains poor [10]. These facts stress the need for developing a recurrence predictive model for HGG, which will assist clinicians in determining and carrying out personalized treatment regimen according to every patient's recurrence rate, and consequently improve the therapeutic effect and reduce treatment-related side effects of HGG patients.

Previous studies have found that some molecular markers were conducive to predict the recurrence of HGG. For example, in the study by Liu et al., increased levels of neuroligin-3 in the deep brain region occurred in pathology situations and might contribute to GBM recurrence [11]. Also, p53 signaling, Notch, Wnt, VEGF, MEK, the hypoxia-related miR-210, the immune-modulatory miR-146b, and other biomarkers with stem-like properties were upregulated in recurrent GBM [12–15]. However, the above studies are limited to predicting recurrence, but no in-depth investigation on the recurrence patterns. Moreover, the vast majority of these predication approaches are implemented mainly through invasive procedures such as repeated venous blood collection, and financially destitute cancer patients have to pay heavy out-of-pocket expenses for detecting some biomarkers. Therefore, it is urgently needed to investigate a cost-effective, painless, and noninvasive method to predict the recurrent patterns for HGG.

In recent years, noninvasive functional imaging techniques are gradually appreciated and applied into the diagnosis, treatment, and OS predication of malignant tumors [16]. Magnetic resonance imaging (MRI), as a cost-effective examination method, could only provide structural information regarding anatomical location of brain tumors and the presence or absence of a disrupted blood-brain barrier in the past. With technological development, advanced MRI modalities are increasingly being used to further characterize GBM in a more comprehensive manner. These include proton magnetic resonance spectroscopy, diffusion imaging, and vascular imaging [17]. In addition, functional MRI and tractography have been increasingly used to identify persuasive cortical and significant tracts to reduce postoperative neurological deficits and improve patient survival [18, 19]. With the supply of biologically relevant functional, haemodynamic, cellular, metabolic, and cytoarchitectural information, advanced standard MRI platforms attract the increasing attention of clinicians and oncologists [20]. Kim et al. [21] effectively discriminated primary CNS lymphoma from GBM in multiparametric MRI using radiomic analyses on regions of interest covering contrast-enhanced tumor, whole tumor, and peritumoral edema (PTE). Henker et al. prospectively evaluated preoperative MRI images from patients harboring a primary supratentorial GBM and illustrated that preoperatively measured necrosis volume was one of the most important radiological features of GBM with a strong influence on OS [22]. However, the potential value of different radiological features obtained by MRI like tumor site, tumor size, and PTE to the recurrence patterns of HGG is still controversial [22], and relevant studies are few.

In this study, we retrospectively analyzed the relationship between the clinical parameters (including age, gender, WHO pathological grade, tumor size, tumor site, clinical treatment regimens, and PTE area) or some molecular markers (Ki-67, MGMT, IDH-1, and p53) and the tumor recurrence patterns identified on MRI in patients pathologically diagnosed with HGG. Furthermore, the effects of these clinical parameters on the recurrence-free survival (RFS) were also studied. Collectively, this study is expected to provide useful information for monitoring recurrence patterns and predicting RFS.

## 2. Materials and Methods

### 2.1. Study Subjects

Between January 1, 2013, and December 31, 2018, patients who fulfilled all of the following inclusion criteria and accepted treatments in the Affiliated Hospital of Xuzhou Medical University were eligible for participation in this single-institution retrospective study.

Inclusion criteria were as follows: (1) pathologically diagnosed as HGG; (2) the PTE characteristics could be accurately judged by MRI images data before surgery; (3) received surgical treatment; (4) at least one MRI scan was obtained after surgery and before recurrence to demonstrate complete surgical resection of the tumor; and (5) tumor recurrence was confirmed by MRI.

Exclusion criteria were as follows: (1) pathologically diagnosed as low grade gliomas; (2) HGG was confirmed by biopsy; and (3) with concomitant malignant diseases.

RFS served as the endpoint in our study, which was measured from the day of operation (equivalent to the day of pathological diagnosis) until the time point of recurrence. RFS beyond the end of the observational period (last follow-up visit) was considered “censored.” All clinical data were taken from the hospital's own records.

The Ethics Committee of the Affiliated Hospital of Xuzhou Medical University approved this study.

### 2.2. MRI-Scans

In order to avoid bias from diverging imaging procedures, preoperative and postoperative MRI scan was performed in-house (obtained on 1.5 mm- or 3.0 mm-Tesla scanners Discovery 750w, GE Healthcare, Milwaukee, WI USA or Ingenia 3.0 T, Philips, Amsterdam, NL). Minimum MRI protocol included axial T1-weighted sequences with and without contrast enhancement, coronal and axial T2-weighted images, or FLAIR sequence for identifying edema and vascularity. Preoperative MRI scan was conducted as early as 1 week before surgery, while postoperative MRI scan was done within 48 h after surgery.

### 2.3. Classifications of Tumor Size, PTE, and Recurrence Patterns on MRI Images

Tumor size was measured as unidimensional largest diameter on axial T2-weighted images, and three groups were defined, including <2 cm, 2-4 cm, and >4 cm.

According to Schoenegger K's criteria [5], PTE was defined as high T2 signal intensity on the tumor margin. On the basis of the distance from the outer edge of abnormally high signal to tumor margin on T2-weighted images, PTE was divided into two levels including <1 cm and ≥1 cm (Figure 1).

The recurrence patterns included the following three types according to Albert et al.'s study [23]: (1) local recurrence (Figure 2(a)): >80% of recurrent contrast-enhancing lesion arose within 2 cm of the original tumor boundary; (2) marginal recurrence (Figure 2(b)): >80% of recurrent contrast-enhancing lesion appeared 2-4 cm away from the original tumor; (3) distant recurrence (Figure 2(c)): >80% of recurrent contrast-enhancing lesion occurred >4 cm from the site of the original tumor. In tumors with multifocal recurrences, they were also defined as “distant recurrence” if any of the foci were >4 cm from the original tumor.

Two experienced oncologists and one experienced radiologist read the MRI images of all patients and identified them according to the above classification criteria. If the results were inconsistent, the three physicians discussed together and finally reached a consensus.

### 2.4. Detection of Immunohistochemical Indicators

Paraffin sections of HGG tissues were dewaxed at 65°C for 4 h by twice 15 min washes with xylene. Then, the sections were rehydrated in graded ethanol to distilled water. Antigen retrieval was carried out by heating the sections in 10 mM citrate buffer (pH 6.0) at 95°C for 30 min, and endogenous peroxidases were blocked by 3% hydrogen peroxide for 10 min. After 30 min blocking with 5% BSA, the sections were incubated overnight at 4°C with the following primary antibodies: Ki-67 (No. 2M-0167, ZSGB-BIO, Beijing, China), MGMT (No. 2M-0461, ZSGB-BIO, Beijing, China), IDH-1 (No. 2M-0447, ZSGB-BIO, Beijing, China), and p53 (No. 2M-0408, ZSGB-BIO, Beijing, China). Then, the sections were incubated with HRP-conjugated secondary antibodies for 30 min at room temperature. On completion of secondary antibody incubation, 3-diaminobenzidine was used for dyeing target proteins and hematoxylin for staining nuclei. Subsequently, the sections were dehydrated and sealed with coverslips. Images were recorded, and 500-1000 tumor cells were counted under 5 microscopic vision fields with an ordinary microscope (Nikon, Japan). The number of Ki-67, MGMT-, IDH-1-, and p53-positive tumor cells were recorded; the positive expression rate (PER) was then calculated by using the formula: PER = number of positive tumor cells in 5 vision fields/total number of tumor cells in 5 vision fields. The interpretation principles of immunohistochemical results are shown in Table 1.

### 2.5. Statistical Analysis

The statistical analysis was done by statistical software SPSS24.0, and quantitative data were presented as mean ± standard deviation (SD). Chi-square test and Fisher test were used to analyze the relationship between recurrence patterns and clinical parameters (age, gender, tumor site, tumor size, WHO pathological grades, clinical treatments, and PTE) and immunohistochemical indicators. COX regression analysis and Log-rank test were employed to explore the influence of these factors on the RFS and to calculate risk ratio (RR) and 95% confidence interval (95% CI). *P* < 0.05 was considered as a statistically significant difference.

## 3. Results

### 3.1. Characteristics of Enrolled Patients

After a rigorous screening process, 77 patients including 38 males and 39 females were included, with a mean age of 48.92 ± 14.135 years old (range: 24-76 years). The characteristics of these enrolled patients are shown in Table 2. The number of HGG patients with large tumors or extensive PTE was relatively large (Tumor size: <2 cm vs. 2-4 cm vs. >4 cm: 6.5% vs. 31.2% vs. 62.3%; PTE: <1 cm vs. ≥1 cm: 27.3% vs. 72.7%).

### 3.2. HGG Patients Were Associated Mostly to Distant Recurrence Pattern

By comparing and analyzing the differences of recurrence patterns in different clinical indicators, we found that almost more than half of the HGG patients had distant recurrence regardless of gender (male: 60.53%; female: 56.41%), age (≤50 years old: 57.89%; >50 years old: 58.97%), WHO pathological grade (III: 54.05%; IV: 62.5%), or previous treatment regimens [surgery: 50%; surgery+ radiotherapy(RT)/chemotherapy and radiotherapy (CRT): 66.67%] (Table 3). Although the number of patients in subgroups of tumor size varied, the rate of distant recurrence in each subgroup was still the highest (Table 3). In addition, tumor location of frontal and parietal lobe (FPL), temporal and occipital lobe (TOL), basal ganglia and thalamus area (BGT), and insular lobe (IL) was associated with incidence rates of distant recurrence ≥ 50%. However, HGG tumor in subtentorial cerebellum and brainstem area (SCB) was more likely to had local recurrence (Table 3). On the whole, the enrolled patients had the highest rate of distant recurrence pattern (Figure 3), and significant differences were existed in subgroups of tumor size (local recurrence vs. distant recurrence: *P* = 0.042, Figure 3(a)) and tumor site (local recurrence vs. distant recurrence: *P* = 0.0020, Figure 3(b)).

### 3.3. PTE Was an Independent Predict Factor of Recurrence Patterns and RFS for HGG Patients

It was worth noting that the recurrence pattern was different in patients with different PTE area, when the PTE was mild (<1 cm), the recurrence pattern tended to be local; in contrast, HGG was more likely to progressed to marginal recurrence or distant recurrence (local recurrence vs. marginal recurrence: *P* = 0.01, local recurrence vs. distant recurrence: *P* = 0.0002, Figure 4(a)). Subsequently, we analyzed the correlation of PTE and RFS; the result showed that the median RFS of the HGG patients with PTE < 1 cm (23.60 months) was obviously longer than those with PTE ≥ 1 cm (5.00 months) (RR = 0.4688, 95% CI: 0.2990-0.7348, *P* < 0.0001, Figures 4(b)–4(d)). The above results indicated that PTE was an independent predict factor of recurrence patterns, and the PTE area was negatively associated with RFS in patients with HGG.

In addition, we also analyzed the effect of other clinical indicators on HGG patients' RFS. The results suggested that age could significantly affect HGG patients' RFS; the median RFS of the HGG patients aged <50 years (8.10 months) was significantly longer than those aged >50 years (6.30 months) (RR = 0.6302, 95% CI: 0.3989-0.9957, *P* = 0.0319, Figure 5). However, the clinical indicators including gender (Figure S1A), age (Figure S1B), WHO pathological grade (Figure S1C), and clinical treatment (Figure S1D) had no significant effect on the RFS of HGG patients.

### 3.4. Expression Level of Ki-67, MGMT, IDH-1, and p53 in HGG Tissues Had No Effect on the Recurrence Patterns

Ki-67, MGMT, IDH-1, and p53 were molecular markers those are routinely detected in clinical diagnosis and treatment, so we further investigated the relationship between the expression levels of them (the representative pictures of different expression levels are shown in Figures 6(a)–6(c)) and the recurrence patterns of HGG patients. Regrettably, all the molecular indicators did not significantly affect the recurrence patterns, because all the *P* values were more than 0.05.

## 4. Discussion

Currently, the standard treatment for newly diagnosed HGG is maximal safe resection, followed by high-dose RT and chemotherapy with temozolomide [24, 25]. In addition, despite these comprehensive therapeutic methods, the vast majority of HGG patients are prone to relapse and progress within a short time. For patients with recurrent HGG after first-line treatment, the alternative treatments are so limited that the management of those population remains challenging [24]. Hence, the accurate prediction of risk and patterns of recurrence in HGG patients is of great concern.

Studies have shown that PTE plays a vital role in the symptoms of GBM patients, which is the main cause of neurological impairment [26]. The severity of PTE, according to existing reports, is significantly associated with the pathological grading of gliomas. PTE on preoperative MRI can serve as an independent prognostic factor in addition to postoperative Karnofsky Performance Scale score, age, and type of tumor resection; patients with major edema have significant shorter overall survival compared to patients with minor edema [1, 27, 28]. However, an ongoing controversy is whether preoperative PTE is a prognostic factor for GBM patients after surgery. Chang et al. confirmed no correlation between PTE volume and GBM recurrence [29]. But in this study, we discovered that PTE was an independent predictor of recurrence patterns and RFS for HGG; the median RFS of HGG patients with mild PTE was significantly longer than those with severe PTE. Our findings were similar to some studies. A retrospective study by Liu et al. revealed that preoperative PTE was an independent prognostic factor for decreased survival in GBM patients [30]. Mummareddy et al. [31] performed segmental volume analysis of preoperative MRI in 210 GBM patients and found that elevated PTE level was associated with decreased survival.

Furthermore, we illustrated that age, gender, WHO pathological grade, and clinical treatment regimens did not statistically affect the recurrence patterns, while gender, WHO pathological grade, clinical treatments, tumor site, and tumor size played negligible roles in changing RFS. We are of the opinion that if more multicenter and large-sample clinical data can be enrolled, some different results may appear.

Previous studies have demonstrated that the expression level of MGMT, Ki-67, and p53 and the mutation status of IDH are closely related with the prognosis of glioma [32–35]. Here, we analyzed the relationship between these molecular indicators and recurrence patterns in HGG patients, but the final results were negative. We suppose that these molecules may only affect the proliferative ability or therapeutic resistance of HGG cells and led to cancer recurrence, but do not play vital roles in the biological process of recurrence patterns.

## Figures and Tables

**Figure 1:** Measurement of PTE by means of MRI T2-weighted images. (a) MRI T2-weighted images showing PTE (peritumoral edema) extending less than 1 cm from the tumor margin; (b) MRI T2-weighted images showing PTE extending more than 1 cm from the tumor margin. Blue circle represented the size of PTE; red circle represented the size of tumor.

**Figure 2:** Recurrence patterns on MRI images. (a) Local recurrence; (b) marginal recurrence; (c) distant recurrence. Red circle represented the tumor.

**Figure 3:** Statistical analysis of the relationship between clinical parameters and recurrence patterns. (a) Tumor size; (b) tumor site. ^∗^*P* < 0.05 vs. local recurrence; ns: no significant. ^∗^*P* < 0.05 vs. local recurrence; ns: no significant.

**Figure 4:** Statistical analysis of the relationship between PTE and RFS. (a) Number of patients with recurrence patterns in different PTE (peritumoral edema) zones. ^∗^*P* < 0.05 and ^∗∗^*P* < 0.01 vs. local recurrence. (b) Swimmers plot of the recurrence-free survival (RFS) for each patient. (c) Scatter plot of the RFS for the two groups; ^∗∗^*P* < 0.01. (d) Kaplan-Meier curve analysis of RFS between the two groups. ^∗∗^*P* < 0.01.

**Figure 5:** Statistical analysis of the relationship between age and RFS. (a) Swimmers plot of the RFS for each patient. (b) Scatter plot of the RFS for the two groups (≤50 years old vs. >50 years old). (c) Kaplan-Meier curve analysis of RFS between the two groups (≤50 years old vs. >50 years old).

**Figure 6:** Expression of Ki-67, MGMT, p53, and IDH-1 in HGG tissues had no effect on the pattern of recurrence. (a) Representative immunohistochemical staining of MGMT, Ki-67, and p53. (b) Representative immunohistochemical staining of IDH-1. (c) Number of patients with the expression of Ki-67, MGMT, p53, and IDH-1 in difference recurrence patterns. ns: no significant.

**Table 1:** The interpretation principles of immunohistochemical results.

Expression level	MGMT	Ki-67	p53	IDH-l
Negative (-)	None	<5%	<5%	None
Weakly positive (+)	<10%	5-25%	5-10%	>0%
Moderate positive (++)	10-30%	26-50%	11-50%	
Strongly positive (+++)	>30%	>50%	>50%	

MGMT: O(6)-methylguanine-DNA methyltranferase (DNA repair enzyme); Ki-67: proliferation marker; p53: molecular marker; IDH-1: isocitrate dehydrogenase (genetic prognosis maker).

**Table 2:** Characteristics of enrolled patients.

Characteristics	*n* (%)
*Gender*	
Male	37 (48.1%)
Female	40 (51.9%)
*Age (years)*	
≤50	38 (49.4%)
>50	39 (50.6%)
*Tumor site*	
FPL	37 (48.1%)
TOL	26 (33.8%)
BGT	6 (7.8%)
IL	3 (3.9%)
SCB	5 (6.5%)
*WHO pathological grade*	
III	37 (48.1%)
IV	40 (51.9%)
*Clinical treatment*	
Surgery	38 (49.4%)
Surgery + RT/CRT	39 (50.6%)
*Tumor size*	
<2 cm	5 (6.5%)
2-4 cm	24 (31.2%)
>4 cm	48 (62.3%)
*PTE*	
<1 cm	21 (27.3%)
≥1 cm	56 (72.7%)

Note: FPL: frontal and parietal lobe; TOL: temporal and occipital lobe; BGT: basal ganglia and thalamus area; IL: insular lobe; SCB: subtentorial cerebellum and brainstem; RT: radiotherapy; CRT: chemotherapy and radiotherapy; PTE: peritumoral edema.

**Table 3:** The incidence rates of local/marginal/distant recurrence in HGG patients with different clinical parameters.

Characteristics	*n*	Local recurrence [*n* (%)]	Marginal recurrence [*n* (%)]	Distant recurrence [*n* (%)]
*Gender*				
Male	38	5, 13.16%	10, 26.32%	23, 60.53%
Female	39	7, 17.95%	10, 25.64%	22, 56.41%
*Age (years)*				
≤50	38	7, 18.42%	9, 23.68%	22, 57.89%
>50	39	5, 12.82%	11, 28.21%	23, 58.97%
*WHO pathological grade*				
III	37	9, 24.32%	8, 21.62%	20, 54.05%
IV	40	3, 7.5%	12, 30%	25, 62.5%
*Tumor size*				
<2 cm	5	0, 0%	1, 20%	4, 80%
2-4 cm	24	7, 29.17%	7, 29.17%	10, 41.67%
>4 cm	48	5, 10.42%	12, 25%	31, 64.58%
*Tumor site*				
FPL	37	5, 13.51%	9, 24.32%	23, 62.16%
TOL	26	2, 7.69%	7, 26.92%	17, 65.38%
BGT	6	1, 16.67%	2, 33.33%	3, 50%
IL	3	0, 0%	1, 33.33%	2, 66.67%
SCB	5	4, 80%	1, 20%	0, 0%
*Clinical treatment regimen*				
Surgery	38	8, 21.05%	11, 28.95%	19, 50%
Surgery+RT/CRT	39	4, 10.26%	9, 23.08%	26, 66.67%
*PTE*				
<1 cm	21	9, 42.86%	5, 23.81%	7, 33.33%
≥1 cm	56	3, 5.36%	15, 26.79%	38, 67.86%
Total	**77**	**12, 15.6%**	**20, 26%**	**45, 58.4%**

Note: FPL: frontal and parietal lobe; TOL: temporal and occipital lobe; BGT: basal ganglia and thalamus area; IL: insular lobe; SCB: subtentorial cerebellum and brainstem; RT: radiotherapy; CRT: chemotherapy and radiotherapy.

## Data Availability

The data used to support the findings of this study are available from the corresponding author upon request.

## Supplementary Materials

Supplementary Materials Supplementary Figure 1: analysis of the relationship between clinical parameters and recurrence patterns. A, Gender; B, age; C, WHO pathological grade; D, clinical treatment regimen. ns: no significant.
